# A comparative analysis of blended learning and traditional instruction: Effects on academic motivation and learning outcomes

**DOI:** 10.1371/journal.pone.0298220

**Published:** 2024-03-04

**Authors:** Rizwan Shoukat, Iskander Ismayil, Qibing Huang, Mohamed Oubibi, Muhammad Younas, Rizwan Munir

**Affiliations:** 1 School of Education, Soochow University, Suzhou, P.R. China; 2 School of Educational Technology, Faculty of Education, Beijing Normal University, Beijing, P.R. China; 3 Smart Learning Institute of Beijing Normal University, Beijing, P.R. China; 4 School of Statistics, Jiangxi University of Finance and Economics, Nanchang, P.R. China; University of Johannesburg, SOUTH AFRICA

## Abstract

The correlational research study aims to examine how blended learning affects academic motivation and achievement. The objectives of the study are to assess students’ opinions on the current level of blended learning, teachers’ practice of blended instruction, the benefits of blended learning, its impact on academic motivation and learning outcomes, and factors influencing blended learning to determine how instructors’ methods influence students’ academic motivation and learning results. The study includes all Bachelor of Science students from various public and private institutions in the Faisalabad Division. Quantitative data from 400 students were collected from four selected institutions. A closed-ended, customized 5-point Likert scale questionnaire was used to collect data. The reliability of the questionnaire was confirmed through expert comments and pilot testing, with a reliability score of (= .97). Data were collected via Google Forms and researcher visits. Descriptive and inferential statistics were employed to analyze the collected data and answer the research questions. The findings of the study indicate that students somewhat agreed with the current blended learning environment, and strongly agreed with variables such as instructors’ blended instruction techniques, the benefits of blended learning, and factors influencing blended learning. Blended learning had statistically significant positive effects on academic motivation and learning outcomes. The findings suggest improving the blended learning environment and instructors’ blended education methods to enhance university students’ academic motivation and learning outcomes.

## 1. Introduction

Previously, teachers and students could only find learning resources in libraries, but with the invention of the Internet, these learning resources can now be found on the Internet. Now teachers and students can study new topics online at home. In recent years, technology has played a greater role in teaching and learning, and now teachers are replacing traditional instructional methods with new ones as technology has become more important in education. One of these innovative methods is known as "blended learning" [1, 2]. Since 1998 when the first surge of web-based learning began, American classrooms have become more diverse, collaborative, and integrated.

Tucker (2012) stated that blended learning "brings traditional classrooms into the tech-friendly 21st century." In addition, blended learning is the most effective approach in the classroom in the 21st century because it encourages students to be innovative, to communicate effectively, think critically, solve problems, collaborate with others, and utilize technology; it also suggests incorporating technology when teaching children 21st-century skills [3]. Blended learning is a formal educational program that combines online and face-to-face instruction. It is a form in which students receive face-to-face instruction, and content is delivered both on campus and online [4]. Blended learning is an educational approach that combines traditional classroom instruction with modern Internet or online instruction [5] and is the best platform for the 21st century because it encourages students to be innovative, to communicate effectively, think critically, solve problems, collaborate with others, and use technology [6]. According to [7], blended learning is a teaching strategy that mixes face-to-face classroom instruction with online learning. This technique can take many different forms, ranging from courses that are mostly online but include some in-person components to programs that are primarily in-person but augment learning with online resources. Blended learning is frequently utilized to give students more flexibility by allowing them to work at their own pace and on their own time. It is explained that blended learning is a teaching method that mixes traditional instruction with online learning activities [8]. This strategy provides students with flexibility, personalization, and active participation, and has been shown to improve their academic performance.

### 1.1. Blended Instruction

Blended instruction is when teachers convey information by applying traditional (face-to-face) training and online teaching methodologies [9]. It mixes face-to-face teaching with online learning. Digital and physical classroom activities are combined to provide an engaging learning experience for students [10, 11]. Blended instruction uses the best of conventional and online learning. In a blended learning environment, students can use videos, books, and interactive tasks outside of class. These digital tools supplement teacher-led education, enabling more personalized and self-paced learning [12]. Blended instruction has been the norm worldwide since 2020 [5]. It incorporates the two teaching approaches using effective instructional design and technology [10, 13, 14]. In addition, it capitalizes on the benefits of both modes of instruction, such as flexible learning time and space, simple access to and sharing of resources, and increased interaction [15]. Some researchers view blended learning as an important method of instruction that circumvents the drawbacks of both traditional classrooms and pure online learning [9, 16].

Blended instruction is a novel method for enhancing teaching, allowing instructors to examine and modify their practices. It benefits from both offline and online learning, and lets students choose when and where to study. Interactive online components stimulate involvement and engagement. Blended education allows students to study subjects independently with instructor assistance [17]. And may be implemented and designed differently in different educational environments. Blended instruction has been studied for its potential to improve student learning and foster 21st-century skills [8].

### 1.2. Benefits of blended learning

According to [18], blended learning benefits students and teachers by allowing personalization of learning. Online components let students customize their learning to their needs and preferences, while online tools and resources give students more learning materials and possibilities than in a traditional classroom. Blended learning also increases student engagement and performance and keeps students engaged and on track. Online assessments and exercises can assist students in identifying areas of weakness and adjusting their learning [11]. Blended courses provide students with greater flexibility by allowing them to access course materials available on websites anytime and study them as needed. Blended learning also allows students more freedom and time to receive feedback [19–21].

### 1.3. Students’ academic motivation

The capacity of a student to achieve either long-term or short-term academic goals can be considered academic motivation. Additionally, it manifests itself as enthusiasm and a positive attitude toward learning. Motivated students are more likely to finish their work and learn new skills. The term “academic motivation” refers to a student’s attitude, tendency, and interest in academic subjects [22–24]. Moreover, it drives behaviors related to academic success, such as students’ effort, workload management, activities, and perseverance [25].

### 1.4. Students’ learning outcomes

Student learning outcomes (SLO) define the expected knowledge, skills, and attitudes students should acquire by the end of a course or program. They ensure that learning objectives are specific, measurable, and aligned with the institution’s main goals. Some common examples of students’ learning outcomes include knowledge acquisition, critical thinking, communication, collaboration, and professionalism [26]. Learning outcomes are the information, skills, and competence a learner gains through a training session, seminar, course, or program [27] and can be categorized as four kinds: cognitive strategy, verbal motivation, motor skills, and attitude.

## 2. Literature review

Blended learning has acquired popularity in higher education due to its potential to improve students’ academic motivation and learning outcomes. It has been studied for its implications for student learning and motivation; for example, [28] evaluated the effects of blended learning on higher education student performance and motivation. According to their study, blended learning greatly increased student academic performance and motivation compared to traditional face-to-face instruction. Similarly, [29] revealed that blended learning improved academic performance, critical thinking, and problem-solving ability. It also enhanced student interest and involvement in learning. Furthermore, [30] evaluated the impact of blended learning on students’ academic motivation and observed that it improved students’ intrinsic motivation, self-efficacy, and interest in course content. A comprehensive review of 77 studies on blended learning revealed that it can improve student achievement, engagement, and satisfaction, especially when online activities are carefully structured to complement and enhance face-to-face education [31]. The review also discovered that blended learning can benefit students from various backgrounds and with various learning requirements because it allows for differentiation, individualization, and self-paced learning. It was reported that blended learning was related to higher levels of student engagement and self-regulated learning compared to traditional learning in a study involving undergraduate engineering students [32].

According to the findings of [33], blended learning substantially influences the academic performance of college students as well as their overall level of satisfaction. [34] discovered increased student engagement and satisfaction in online courses using blended learning. Examination of the impact of blended learning on the academic performance of college students enrolled in a business statistics course discovered that students who participated in the blended learning program performed much better than those who just received traditional face-to-face education [35]. Moreover, [3] examined the effect of blended learning on students’ reading comprehension skills and discovered that students who participated in a blended learning program improved their reading comprehension more than those who only received standard classroom-based training.

A previous study examined how blended learning motivated Korean college students to succeed. According to the study, the blended learning strategy motivated and controlled students and improved their grades [36]. Flipped classrooms were found to influence Korean college students’ academic motivation. The flipped classroom strategy increased their self-efficacy and competence, which enhanced their school performance and motivation [37]. [38] examined how blended learning motivated Jordanian college students to succeed, and found that it increased student self-motivation and satisfaction with learning. Blended learning also motivated Chinese college students to succeed, and the blended learning strategy improved students’ self-esteem, motivation to learn independently, and perceptions of their learning [39].

In addition, several other studies demonstrated that blended learning positively affects learners’ learning attitudes [40–43] such as developing their learning motivation, increasing their flexibility and self-confidence [44–46], and improving their ability and attitude towards work in groups [48]. Therefore, blended learning improves engagement and enhances the student’s learning experience [48–50]. Another way that blended learning empowers students is by improving their communication skills, thinking skills, problem-solving skills, and technology literacy skills.

Based on the outcomes of the research, blended learning appears to have the potential to be an effective technique for motivating students. It may also help students build their self-motivation, self-control, and self-confidence, which may help them achieve better learning outcomes. It can effectively improve students’ academic motivation and performance, and it can help them engage more deeply with the material and reach higher levels of accomplishment by combining the benefits of face-to-face education with the flexibility and personalization of online learning.

On the other hand, the impacts of blended learning on academic motivation and learning outcomes are not completely known; hence, additional study is necessary in this area. For example, it was discovered that blended learning positively influenced students’ academic motivation in higher education, but that this effect was contingent on the level of interaction between students and instructors [51]. The research demonstrates that by combining traditional and online training benefits, blended learning can effectively and efficiently improve students’ academic achievement. However, it is critical to ensure that the design and implementation of blended learning are founded on good pedagogical principles and consider the learners’ unique context and needs.

### 2.1. Statement of the problem

Blended learning was possible before the recent coronavirus outbreak, but now it is necessary. In addition, due to the rapid technological advancements in recent years, many businesses and public and private educational institutions are beginning to recognize the advantages of adopting a blended learning approach. In the existing literature, studies have yet to be carried out on the effect of a blended learning approach on Pakistani university students’ academic motivation and learning outcomes. This study will fill this gap by exploring the effect of blended learning on students’ academic motivation and learning outcomes and the impact of teachers’ practices on students’ academic motivation and learning outcomes in Pakistani higher education.

### 2.2 Research question and hypotheses

The research questions and hypotheses developed for the current study are as follows:

1. What are students’ opinions on the current environment for blended learning and teachers’ practice of blended instruction?
2. What is the effect of blended learning on students’ academic motivation and learning outcomes, and what factors influence blended learning?

This study is based on seven general hypotheses:

Hypothesis 1 (H1): Blended learning has a positive and significant impact on students’ academic motivation.

Hypothesis 2 (H2): Blended learning positively and significantly impacts students’ learning outcomes.

Hypothesis 3 (H3): Blended learning positively and significantly impacts teachers’ practices.

Hypothesis 4 (H4): Teachers’ practices positively and significantly impact students’ academic motivation.

Hypothesis 5 (H5): Teachers’ practices positively and significantly impact students’ learning outcomes.

Hypothesis 6 (H6): Teachers’ practices mediate the relationship between blended learning and students’ academic motivation.

Hypothesis 7 (H7): Teachers’ practices mediate the relationship between blended learning and students’ learning outcomes.

## 3. Materials and methods

The primary aim of the current study was to investigate the effects of blended learning on students’ academic motivation and learning outcomes. The School of Education of Soochow University’s ethical committee review board reviewed and approved the study, and the participants were provided with an explanation regarding the objectives of the study. Also, reassurance was given to participants that their comments would be utilized exclusively for research purposes. The participants in our study’s survey are acknowledged, and we appreciate all the researchers who helped with data gathering and processing.

According to the said aim, this study utilized a correctional investigation. All the Bachelor of Science (BS) program students studying in public and private sector universities of the Faisalabad Division of Pakistan constituted the population of the current investigation. The targeted population comprised all the BS program students of four universities (two public and two private). A sample comprising 400 students for quantitative data collection was selected through a simple random sampling method from the four universities, and data were collected from January to July 2023. An adapted instrument in the form of a questionnaire developed by [52] was utilized for quantitative data collection from university students. The validity and reliability of the students’ questionnaire were established by obtaining expert opinions from the supervisor and experts. Later on, the researcher conducted a small-scale pilot study. The collected data in the pilot study were measured in SPSS, and a scale reliability test was used to calculate the inter-consistency of the instrument through Cronbach’s alpha value. Cronbach’s alpha (α = .97) showed that the instrument is trustworthy and acceptable for data gathering on a large scale. Later, with the help of a research assistant and Google Forms, the data were collected. Descriptive and inferential statistics were used to examine the connection between independent and dependent variables in SPSS (Version 26). Additionally, structural equation modeling (SEM) was performed for hypotheses assessment. Structural equation modeling is a robust multivariate statistical tool based on covariance statistics. Below are the findings of the data analysis and research model that were utilized for this study.

### 3.1. Research framework

Given the above, a conceptual framework was developed as shown in Fig 1.

**Fig 1:** Research framework.

### 3.2. Ethical considerations

The existing study was conducted in the division of Faisalabad of Pakistan. The researcher followed ethical guidelines during the study. A permission letter was obtained from the supervisor and members of the Ethics Committee of the School of Education at Soochow University, Suzhou, Jiangsu, China. This study involved the completion of a questionnaire that comprised statements related to blended learning, teachers’ practices, benefits, academic motivation, learning outcomes, and factors that influence blended learning. The participants of the study comprised university students studying in the BS program at four universities in Faisalabad division. Moreover, before the collection of data, it was ensured that all participants were aware of the objectives of the study, that the participant consent form was attached to the instrument, and that all of the necessary approvals had been obtained. The collected information was utilized only for academic purposes and was kept confidential.

## 4. Data analysis and results

Descriptive analysis was conducted to compute mean scores and standard deviations. The students’ perceptions of the study’s variables were evaluated based on the criteria established in the literature [2]. The adopted criteria are as follows: Criteria to assess students’ level of agreement/disagreement with the current environment of blended learning, teachers’ practices, benefits, and effects on students’ academic motivation and learning outcomes (see Table 1).

**Table 1:** Descriptive statistics.

No.	Mean Score	Level of Agreement
1	Less than 1.8	• Very Low
2	1.8 to 2.6	• Low
3	2.6 to 3.4	• Moderate
4	3.4 to 4.2	• High
5	4.2 and above	• Very High

Table 2 demonstrates the students’ opinions on each factor of blended learning. Results show that students had a moderate level of agreement with the factor of the existing environment of blended learning (Mean = 3.34, *SD* = 1.044), while there was a higher level of agreement with the factor of teachers’ practices of blended instruction (Mean = 3.54, *SD* = 1.007).

**Table 2:** Students’ opinions on each factor of blended learning (*N* = 400).

S. No.	Factors	Mean	*SD*	Level of Agreement	Rank
1.	The Environment of Blended Learning	3.34	1.044	-Moderate	7
2.	Teachers’ Practices of Blended Instruction	3.54	1.007	-High	4
3.	Benefits of Blended Learning	3.60	0.919	-High	1
4.	Effects of Bended Learning on Students’ Academic Motivation	3.59	0.891	-High	2
5.	Effects of Blended Learning on Students’ Learning Outcomes	3.54	0.881	-High	3
6.	Factors Influencing Blended Learning	3.52	0.907	-High	5

Table 3 shows the statistical results that occurred during the execution of the *t* test. It was performed to compare blended learning characteristics by student gender. Results show that female students had better agreement with the blended environment (Mean = 3.4515, *SD* = .64019) while male students had less agreement with the blended environment (Mean = 3.2595, *SD* = .76606), (*p*-value = .007 < .05 level).

**Table 3:** Factor-wise comparisons of blended learning based on students’ gender.

Factors	Gender	*N*	Mean	Std. Deviation	*p*-value
Environment	Male	200	3.2595	.76606	.007
	Female	200	3.4515	.64019	
Teaching_ Practices	Male	200	3.4215	.91178	.001
	Female	200	3.6685	.57786	
Benefits	Male	200	3.5230	.85987	.026
	Female	200	3.6895	.60421	
Academic_ Motivation	Male	200	3.4920	.82489	.004
	Female	200	3.6995	.58176	
Learning_ Outcomes	Male	200	3.4533	.83595	.011
	Female	200	3.6408	.62296	
Factors Influencing_ BL	Male	200	3.4860	.83480	.288
	Female	200	3.5650	.63671	

The statistical results reported in Table 4 show the mean scores, standard deviation, alpha value, and relationship statistics among the variables. The study included four variables: blended learning (IV), practices (M), academic motivation and learning outcomes (DV). The reliability scores (Cronbach’s alpha) for each research instrument show that the internal consistency of the scales met the alpha threshold suggested by Nunally (1978). Moreover, the correlation analysis estimates the strengths and weaknesses of relationships among variables. In this study, all variables had positive and statistically significant correlations. Furthermore, correlation demonstrates that there is no issue of overlapping or multicollinearity among variables.

**Table 4:** Mean scores, std. deviations and alpha values.

Variables	Mean	*SD*	Α	1	2	3	4
Blended Learning	3.34	1.044	.86	.701**			
Practices	3.54	1.007	.92		.728**		
Academic Motivation	3.59	.891	.94			.709**	
Learning Outcomes	3.54	.881	.91				.656**

### 4.1. Structural equation modeling (SEM) Results

The theoretical framework shows the four variables to be studied. Blended learning is considered an endogenous factor which was estimated with seven measured items. The students’ academic motivation and learning outcomes were taken as the exogenous factors. The factors of academic motivation and learning outcomes were estimated with five measured items each. The framework uniquely illustrates teachers’ practices as a mediating factor between blended learning, academic motivation, and learning outcomes. Structural equation modeling (SEM) is one of the latest multivariate statistical approaches that helps to provide robust statistical results. It essentially includes measurement and structural models and is a more restricted version of multivariate statistics that gives valid and non-spurious path coefficients. Accordingly, in this research CB-SEM was adopted as a multivariate statistical tool for both measurement and structural analysis.

### 4.2. Confirmatory factor analysis

Fig 2 demonstrates the confirmatory factor analysis (CFA) for the measurement part of the model. The CFA results confirmed that each construct had its own explaining power that did not overlap with other constructs. The covariance statistics represent that each construct is in line with their respective measurement items. Furthermore, the validities such as convergent and discriminant validity were also observed and were found to be consistent with the measured items. The convergent validity composite reliability (CR) was more than .70 and the average variance extracted (AVE) was more than .50 for each of the constructs, thus meeting the thresholds for convergent validity. In addition, to ensure that constructs did not overlap with others, discriminant validity was also established. For discriminant validity, it was seen that the squared multiple correlation coefficient (SMCC) for each of the factors was not greater than the AVE score of the restive construct. The CFA helps to identify the model and its goodness of fit (Gof) through fit indices. The fit indices such as CMIN/*df*, CFI, TLI, PCFI, NFI, and RMSEA were all found to be under the minimum suggested thresholds. Afterwards, the hypotheses assessment was made by assessing the structural analysis of SEM.

**Fig 2:** CFA.

**Fig 3** shows the outcomes for Hypotheses 1 and 2. H1 stated that blended learning has a positive and significant impact on students’ academic motivation. In this regard, the model output showed that blended learning had a .58 or 58% positive effect on students’ academic motivation at a 0.01 level of significance. The factor loading for blended learning was estimated with BL1, BL2, BL3, BL4, BL5, BL6 and BL7 and academic motivation with AM1, AM2, AM3, AM4, and AM5. All item loadings were suitable enough and were identified in the CFA model. On the other hand, H2 of this study stated the positive and significant impact of blended learning on students’ learning outcomes. In this regard, the statistical results showed that blended learning had a .62 or 62% positive effect on students’ learning outcomes at a 0.01 level of significance. The item loading for learning outcomes was suitable enough. According to the above-mentioned results, hypotheses 1 and 2 were supported.

**Fig 3:** Confirmatory factor analysis (CFA-modified).

### 4.3. Mediation analysis

This research adapted the mediation mechanism of Barron and Kenny (1986). According to this mechanism the mediation can be proved or disproved based on the criterion of Path-C, Path-A, Path-B, and Path-C’. In Fig 4, Path-C for blended learning, academic motivation, and learning outcomes was proved, and so H1 and H2 were retained. Now, Path-A and Path-B with Path C’ were assessed from the statistical outcomes of Fig 3. According to Path-A, hypothesis 3 was assessed. It stated that blended learning has a positive and significant impact on teachers’ practices, and the results confirmed that blended learning had a .66 or 66% positive impact on teachers’ practices at the 0.01 level of significance. Furthermore, Path B was assessed for both outcome factors; therefore, hypotheses 4 and 5 were examined to confirm the positive and significant impact of teachers’ practices on academic motivation and learning outcomes. In this connection, the statistics showed that teacher practices had a .49 positive impact on academic motivation and a .54 positive impact on learning outcomes at the 0.01 level of significance. Hence, H3, H4, and H5 were consistent with the results in the previous literature. Lastly, the induction of teachers’ practices as a mediator was assessed with Path-C’. In this regard, hypotheses 6 and 7 stated that teachers’ practices mediate the relationship between blended learning, academic motivation, and learning outcomes. Fig 3 shows that after the induction of the mediator, Path-C’ showed the indirect impact of blended learning on academic motivation with .22. Previously, Path-C (Fig 2) showed an impact of .58, so after induction of teachers’ practices as the mediating factor, the beta coefficient was reduced to .22 and became insignificant, which confirms that teachers’ practices had a mediating effect on the relationship between blended learning and students’ academic motivation. Adding to that, teachers’ practices had a mediating effect on the relationship between blended learning and students’ learning outcomes, reducing Path = C’ to .18 and making it insignificant. As per the given results in Fig 5, hypotheses 6 and 7 were also accepted and were consistent with the literature. The results of the Goodness of Fit (GoF) indices were CMIN/*df* = 1.23, CFI = .930, GFI = .956, AGFI = .944, TLI = .890, RMSEA = .032.

**Fig 4:** Hypotheses assessment (H1 and H2).

**Fig 5:** Mediation analysis of teachers’ practices.

## 5. Discussion

This study found a strong positive relationship between blended learning and academic motivation (r = .709). This finding is aligned with the study findings of [53–55] as they also emphasized the effect of a blended learning environment on enhancing student motivation and engagement in the academic setting, and provided a blended learning motivation model for instructors. In addition, according to [56–58], there are several reasons why the blended learning environment and academic motivation are positively correlated based on the level of students and the environment and the use of attractive teaching tools. First, a dynamic and interactive learning environment is produced by employing numerous technology tools, including learning management systems, multimedia materials, and online collaboration platforms. These tools support peer contact, active involvement, and knowledge production, all of which have been shown to improve learning outcomes and motivation. Following [59, 60], the blended learning environment allows students to engage in self-directed learning. Students may take charge of their education, establish objectives, track their progress, and reflect on their learning experiences using online platforms and tools. As a result of these self-directed learning opportunities, students become intrinsically motivated since they see themselves as active participants in their education. The investigation reported a statistically significant positive relationship between blended learning and students’ learning outcomes (r = .656). The results showed that these two variables had a statistically significant and favorable relationship. The reported results are consistent with other research conducted by [61–63] that highlighted the beneficial effects of blended learning on raising academic achievement and learning outcomes for students, and the reported positive outcomes suggest that the combination of traditional and online learning modalities in blended learning fosters a deeper understanding of the subject matter. The accessibility of digital resources and the ability to revisit online materials contribute to reinforcing key concepts and promoting retention. According to [64], incorporating technology and online resources into the traditional classroom setting allows students to engage in interactive and self-directed learning, which can improve their knowledge, understanding, and recall of course information. According to the findings, there is a statistically significant and positive correlation between the practices of instructors’ and students’ levels of academic motivation (r = .728), and between the practices of teachers’ and students’ levels of learning outcomes (r = .701). The findings align with earlier research highlighting the importance of effective instructional practices in blended learning environments for enhancing students’ motivation and academic achievement [65, 66].

Moreover, according to [67, 68], mixed teaching helps children learn to study independently, and students have the autonomy to learn independently in online and blended education. According to [69–71], online tools, interactive assignments, and self-paced learning empower students to establish objectives, measure progress, and take ownership of their learning. Freedom and control over learning motivate learners, boost their self-esteem, and improve their academic performance. The freedom and control afforded to students in this context have several positive outcomes. Firstly, having the flexibility to choose learning objectives allows students to tailor their educational experience to align with their interests and goals [72]. This personalized approach fosters a sense of autonomy and agency, contributing to a more engaging and meaningful learning experience. Moreover, the ability to measure progress allows students to gauge their success, fostering a sense of accomplishment and motivation. When students have a clear understanding of their academic advancements, it not only boosts their self-esteem but also serves as a powerful motivator to continue striving for excellence [73].

The notion of taking ownership of learning implies that students become active participants in their educational journey. This sense of responsibility can lead to increased commitment and dedication to the learning process. As a result, students are more likely to be invested in their studies, contributing to improved academic performance [74]. The study highlighted that when teachers use technology in blended learning, they can give students immediate feedback, special help, and customized learning experiences [75]. With online tools and learning management systems, teachers can keep track of their students’ success, figure out where they need to improve, and help them in those areas [76]. This kind of personalized help gets students more interested in learning and also helps them improve their academic motivation and learning outcomes.

## 6. Conclusions

Based on the above results, it was concluded that the students had a moderate level of agreement with the factor of the existing environment of blended learning and that they had a higher level of agreement with the factor of teachers’ practices of blended instruction. Students also had higher levels of agreement with the benefits of blended learning and with the factor of the effects of blended learning on their academic motivation and learning outcomes. This exploration exposed that students had a higher level of agreement with the factors that influence blended learning, such as lack of availability of quality technological infrastructure, ineffective instructional design, lack of teachers’ training to deliver blended learning courses, lack of students’ readiness and technical skills, and lack of university administration, technical, and financial support. In addition, this investigation discovered a statistically significant relationship between blended learning and students’ academic motivation and learning outcomes. It was also discovered that teachers’ practices had a statistically significant positive relationship with students’ academic motivation and learning outcomes.

Moreover, SEM results concluded that blended learning positively and significantly impacted student academic motivation. In this regard, the model output discovered that blended learning had a .58 or 58% positive impact on students’ academic motivation. There was a positive and significant effect of blended learning on students’ learning outcomes. In this regard, the statistical results indicated that blended learning had a .62 or 62% positive impact on students’ learning outcomes. It also discovered that blended learning had a positive and significant impact of .66 or 66% on teachers’ practices and that teacher practices had a .49 or 49% positive impact on academic motivation. The outcomes of SEM showed that teacher practices had a .54 or 54% positive impact on learning outcomes at a 0.01 significance level, and it was revealed that teachers’ practices mediated the relationships between blended learning and students’ academic motivation, and between blended learning and students’ learning outcomes.

### 6.1. Limitations and future research

The current study focused on examining students’ perceptions of blended learning, including its benefits and impacts on their academic motivation and learning outcomes, within the context of four universities (comprising two public and two private institutions) in the Faisalabad Division of Pakistan. This research particularly emphasized the factors influencing the effectiveness of blended learning in these settings. However, a more comprehensive investigation could be undertaken by exploring additional variables related to student performance and extending the research to include universities in other regions of Pakistan. Such an expanded study could provide deeper insights into the broader applicability and potential variations of blended learning effectiveness across different educational and cultural contexts in Pakistan.

### 6.2. Implications

The findings of this study demonstrate the effectiveness of blended learning as a transformative educational approach in enhancing university students’ academic motivation and learning outcomes. This comprehensive assessment reveals that specific components of blended learning, notably the integration of interactive online resources, flexible scheduling, and personalized face-to-face instruction, play a pivotal role in this improvement. Students reported heightened engagement and better comprehension when exposed to these blended learning strategies, marking a significant improvement over the traditional lecture-based method. Moreover, the study’s comparative analysis between blended and traditional learning models highlights a clear preference for the former, with notable increases in student participation, retention rates, and overall satisfaction. These insights are crucial for educational institutions aiming to adapt to evolving pedagogical landscapes and meet the diverse learning needs of students.

## Supporting information

S1 Checklist Human participants research checklist. (DOCX)

S1 Data (XLSX)

S1 Questionnaire (PDF)
